RETRACTED

# miR-19a-3p Promotes Tumor-Relevant Behaviors in Bladder Urothelial Carcinoma via Targeting THBS1

**DOI:** 10.1155/2021/2710231

**Published:** 2021-10-28

**Authors:** Gang Xu, Junlong Li, Lihang Yu

**Affiliations:** Department of Urology, Shaoxing People's Hospital (Shaoxing Hospital), Zhejiang University School of Medicine, Shaoxing City, Zhejiang Province 312000, China

## Abstract

**Objective:**

miR-19a-3p is widely increased in several cancers and can be used as an oncogenic factor in these cancers. However, the molecular mechanism of miR-19a-3p in bladder urothelial carcinoma (BLCA) is still open. So, the study was aimed at exploring the mechanism of miR-19a-3p in BLCA cells.

**Methods:**

Bioinformatics analysis was employed to find the differential miRNAs and mRNAs, and the target miRNA and mRNA were determined. Real-time quantitative PCR was used to evaluate miR-19a-3p and THBS1 levels in human urethral epithelial cells and BLCA cells. Western blot was carried out to assay protein expression of THBS1 in human urethral epithelial cells and BLCA cells. Behaviors of BLCA cells were detected through cellular functional assays. Dual-luciferase gene assay was conducted to validate the binding of miR-19a-3p and THBS1.

**Results:**

miR-19a-3p was increased in BLCA cells, while THBS1 was less expressed in BLCA cells. The miR-19a-3p functions as an oncogene in BLCA. THBS1 was a target of miR-19a-3p, and it could reverse the promotion of miR-19a-3p on cell malignant behaviors in BLCA.

**Conclusion:**

miR-19a-3p facilitates cell progression in BLCA via binding THBS1, which may be an underlying therapeutic target for BLCA treatment.

## 1. Introduction

According to cancer statistics in China, the mortality and morbidity of bladder cancer rank first among all malignant tumors in the urinary system, which seriously reduces the quality of life of human beings [1]. Bladder cancer can be divided into the bladder epithelial tumor and bladder nonepithelial tumor, of which the bladder epithelial tumor accounts for 95%-98% [2–4]. In bladder epithelial tumors, bladder urothelial carcinoma (BLCA) is the dominant one, accounting for about 90% of bladder epithelial tumors [2–4]. Currently, surgery is dominant for BLCA management, but a high recurrence rate with frequent local infiltration and distant metastasis of BLCA leads to unsatisfactory treatment effects on patients with advanced BLCA [5, 6]. Therefore, in order to find more effective treatments for BLCA, we urgently need to illustrate the mechanism involved in the occurrence and development of BLCA, thereby finding potential molecular therapeutic targets for BLCA patients at the molecular level.

In recent years, with the in-depth research on microRNA (miRNA), it has been confirmed that miRNA is often dysregulated in tumors, including BLCA in this study. miR-19a-3p is implicated in the progression of varying diseases [7–9]. For example, Li et al. [10] confirmed that the miR-101-3p level is increased in BLCA. By observing the miR-99a-5p level in BLCA cells SV-Huc-1, 5637, and T24, Tsai et al. [11] manifested that miR-99a-5p presented low expression in both the 5637 and T24 cell lines. At the same time, researchers further found that the dysregulated miRNA also has the function of regulating BLCA progression. For example, Song et al. [12] displayed that decreased miR-199a-5p can induce BLCA by directly regulating MLK3. Zhang et al. [13] confirmed that the miR-30a level is decreased in BLCA, and miR-30a hinders the progression of BLCA cells. Therefore, based on the regulatory effect of miRNA on the progression of BLCA, numerous miRNAs are promising molecular therapeutic targets of BLCA, such as miR-133b [14], miR-429 [15], and miR-331-3p [16]. However, it is still unknown whether miR-19a-3p is dysregulated in BLCA and whether it has the function of regulating the progression of BLCA.

RETRACTED

We confirmed in this research the dysregulation of miR-19a-3p in BLCA and observed the impact of miR-19a-3p on BLCA progression through biological function experiments to identify whether miR-19a-3p can regulate the progression of BLCA. Finally, the molecular mechanism of miR-19a-3p was probed in BLCA so as to lay the groundwork for miR-19a-3p as a molecular target for BLCA patients.

## 2. Materials and Methods

### 2.1. Bioinformatics Methods

Datasets of mRNA expression (normal: 19; tumor: 408) and miRNA expression (normal: 19; tumor: 412) related to BLCA were obtained from TCGA database. miRNA and mRNA data were subjected to differential analysis by using the R package “edgeR,” with normal samples as controls, ∣logFC | >2, and adjusted *p* value < 0.05 as selection criteria. The downstream mRNAs with binding sites of the target miRNA were predicted through starBase, TargetScan, miRTarBase, miRWalk, and miRDB databases. The decreased mRNA was selected as the likely target mRNA of miR-19a-3p.

### 2.2. Cell Culture

Human urethral epithelial cell line SV-Huc-1 (No. 3131C0001000700169) and BLCA cell lines T24 (No. 3131C0001000700055), 5637 (No. 3131C0001000700001), and RT4 (No. 3131C0001000700225) were all accessed from Cell Resource Center, Shanghai Institutes for Biological Sciences, Chinese Academy of Sciences. SV-Huc-1 cells were cultivated in an F12K medium added with 10% fetal bovine serum (FBS). T24 and 5637 cells were cultivated in a Roswell Park Memorial Institute- (RPMI-) 1640 medium supplemented with 10% FBS. RT4 cell lines were cultivated in McCoy's 5A medium with 10% FBS. Then, all the media were nurtured in moist incubators under routine conditions.

RETRACTED

### 2.3. Cell Transfection

The miR-19a-3p-mimic, oe-THBS1, and corresponding control obtained by RiboBio Company were utilized for transfection by a Lipofectamine 2000 reagent. Two days later, cells were collected for preparation.

### 2.4. qRT-PCR

A TRIzol reagent (Invitrogen, Carlsbad, CA, USA) was implemented for total RNA isolation. Then, a PrimeScript RT kit (Takara, Tokyo, Japan) was introduced for cDNA synthesis. A qRT-PCR kit (TransGen Biotech, Beijing, China) was implemented for relative expression assessment of miR-19a-3p and THBS1, with U6 and GAPDH as controls, respectively. The primer sequence is shown in Table 1.

### 2.5. Western Blot

Detail procedures of Western blot were done following the method described in [17]. Primary antibodies included rabbit anti-THBS1 (18304-1-AP, 1 : 1000) or rabbit anti-GAPDH (10494-1-AP1, 1 : 5000) purchased from Proteintech, China. The secondary antibody IgG H&L (HRP) (ab6721, 1 : 8000) was purchased from Abcam, UK.

### 2.6. Cell Counting Kit-8 (CCK-8) Experiment

Following digestion and mixing, T24 cells in the logarithmic growth phase were placed in 96-well plates (2 × 10^4^). A CCK-8 reagent was dropped into the well every 24 h from 0 h to 72 h, and cells were incubated for 2 h. Finally, an enzyme immunoassay analyzer (Bio-Rad, California, USA) was introduced to detect absorbance at 450 nm.

### 2.7. Colony Formation Assay

Cells (4 × 10^2^) were maintained for 2 weeks after being inoculated to 6-well plates. After visible spots appeared in the well, the medium was discarded and 4% paraformaldehyde was utilized for fixing. Then, cells were stained with crystal violet. The number of cell clones in wells was counted after drying.

### 2.8. Wound Healing Assay

After conventional, by trypsin digestion, mixing of T24 cells at the logarithmic phase, 8 × 10^5^ cells were placed in 6-well plates. When they grew to 90%, a monolayer of cells was scraped manually with a sterile pipette tip (200 *μ*L). Then, detached cells were rinsed off with PBS, and remained cells were added with an FBS-free culture medium for culture. The wound was photographed with an inverted microscope (Olympus Corporation, Japan) at 0/48 h after the wound was generated. The cell migration rate was computed.

### 2.9. Transwell Invasion Assay

A Transwell chamber (EMD Millipore, Billerica, MA, USA) was used for invasion assessment of T24 cells. Then, 2 × 10^5^ T24 cells were placed into the top of the insert precoated with Matrigel (BD Biosciences, USA) and the medium+10% FBS was added into the lower chamber. After being maintained in a moist incubator under routine conditions for 24 h, cells that failed to invade were discarded, while cells that invade to the other side were fixed 10 min with 4% paraformaldehyde and stained 30 min with crystal violet. Five fields in each well were randomly selected after drying, and cells were counted under an inverted microscope.

RETRACTED

### 2.10. Dual-Luciferase Reporter (DLR) Assay

Binding sites of miR-19a-3p and its target mRNA were identified by TargetScan. From GenePharma, luciferase reporter vectors (THBS1-Mut, vector containing mutant THBS1; THBS1-Wt, vector containing wild-type THBS1) were accessed. The purchased THBS1-Wt vector or THBS1-Mut vector was cotransfected, respectively, to T24 cells with miR-19a-3p-mimic or NC-mimic. After 48 h, firefly and Renilla luciferase activities were assayed on the luciferase assay system (Promega, USA).

### 2.11. Statistical Analysis

Data were presented as mean ± SD. Statistical analyses were processed on GraphPad Prism 6 software, and comparison between groups was estimated with Tukey's test. Statistical significance was considered to be represented by a value of *p* < 0.05.

## 3. Results

### 3.1. miR-19a-3p Is Upregulated in BLCA

We used edgeR differential analysis to analyze miRNAs differentially expressed in BLCA tissue and normal tissue from TCGA database and finally obtained 144 differentially expressed miRNAs (Figure 1(a)). miR-19a-3p regulates the progression of gastric cancer and liver cancer [8, 18]. Therefore, among these differential miRNAs, we selected miR-19a-3p with noticeably increased expression in BLCA tissue as the study object. The specific level of miR-19a-3p in BLCA and normal tissue samples in TCGA database is shown in Figure 1(b). In order to verify the analysis result in TCGA database, we assayed the miR-19a-3p level in T24, 5637, RT4, and normal cells via qRT-PCR. The miR-19a-3p level was notably increased in T24, 5637, and RT4 cells (Figure 1(c)), and the miR-19a-3p level in T24 cells was the most significant. Therefore, further experiments were conducted in T24 cells. Through the above studies, we proved that the miR-19a-3p level was indeed elevated in BLCA.

### 3.2. miR-19a-3p Promotes the Malignant Progression of BLCA Cells

To probe into the possible role of miR-19a-3p in BLCA, we transfected miR-19a-3p-mimic into T24 cells and confirmed by qRT-PCR that it could overexpress miR-19a-3p in T24 cells (Figure 2(a)). CCK-8 and colony formation assays disclosed marked facilitation of the forced miR-19a-3p level on proliferation and colony formation properties of T24 cells (Figures 2(b) and 2(c)). In addition, the experimental results of wound healing and cell invasion assays also disclosed a similar impact on migratory and invasive properties of T24 cells (Figures 2(d) and 2(e)). The results of these cell biological function experiments fully displayed that miR-19a-3p affected the phenotype of BLCA cells.

RETRACTED

### 3.3. THBS1 Is a Downstream Target of miR-19a-3p

In order to probe into the molecular mechanism of miR-19a-3p in BLCA, we introduced edgeR differential analysis to analyze the differentially expressed mRNAs in BLCA and normal tissue samples. 1595 differentially expressed mRNAs were obtained (835 upregulated and 760 downregulated) (Figure 3(a)). Then, we screened mRNAs with binding sites of miR-19a-3p using 5 gene databases (miRTarBase, miRDB, TargetScan, starBase, and miRWalk) and intersected the screened mRNAs with 835 downregulated mRNAs. Finally, only one mRNA (THBS1) was obtained (Figure 3(b)). The specific level of THBS1 in BLCA and normal tissue samples in TCGA database is plotted in Figure 3(c). For validation, we firstly detected the THBS1 level in SV-Huc-1 and BLCA cells by qRT-PCR and Western blot. mRNA and protein expression of THBS1 in T24, 5637, and RT4 cell lines was prominently decreased (Figure 3(d)). Then, we observed whether miR-19a-3p could target THBS1 by DLR assay. The result showed that miR-19a-3p-mimic could significantly decrease the luciferase activity of the THBS1-Wt reporter gene (Figure 3(e)). Finally, qRT-PCR and Western blot were introduced to observe the impact of overexpression of miR-19a-3p on the expression level of THBS1 in T24 cells. We found that overexpression of miR-19a-3p notably weakened the THBS1 level in T24 cells (Figure 3(f)). Through these experiments, we fully verified that THBS1 was the downstream mRNA of miR-19a-3p.

### 3.4. miR-19a-3p Fosters Malignant Phenotypes of BLCA Cells through Binding THBS1

Although we confirmed that THBS1 was a downstream target of miR-19a-3p in Section 2.3, whether miR-19a-3p could facilitate the progression of BLCA through THBS1 is still open. We then designed a rescue experiment for observation. Firstly, we divided the experiment into the NC-mimic+oe-NC group, miR-19a-3p-mimic+oe-NC group, and miR-19a-3p-mimic+oe-THBS1 group and transfected them into T24 cells. qRT-PCR and Western blot results as depicted in Figure 4(a) showed that oe-THBS1 transfection could partially rescue the repressive impact of miR-19a-3p on the THBS1 level in T24 cells. Besides, THBS1 was observed to markedly reduce the promoting impact of miR-19a-3p on proliferative, migratory, and invasive abilities of T24 cells (Figures 4(b)–4(e)). Together, we summed up that miR-19a-3p exacerbated BLCA cell malignant progression via binding THBS1.

RETRACTED

## 4. Discussion

miR-19a-3p is a member of the miR-17-92 gene cluster and is located on human chromosome 13q31.3 [19]. Previous studies had shown that the miR-19a-3p level is increased in varying cancers, containing gastric cancer [8], breast cancer [20], and prostate cancer [21]. Moreover, the miR-19a-3p level is also increased in exosomes isolated from the urine sediment of patients with bladder cancer [22]. We displayed that miR-19a-3p was also increased in BLCA tissue in TCGA database by using the bioinformatics analysis. Meanwhile, we authenticated the increased miR-19a-3p level in BLCA cells. Increased miR-19a-3p can also facilitate the development of multiple cancers. For instance, miR-19a-3p regulates the Wnt/*β*-catenin signaling pathway by targeting FoxF2, thus promoting malignant behaviors of colorectal cancer cells [23]. miR-19a-3p promotes HCC cell growth via the PIK3IP1/AKT signaling pathway [18]. By cellular functional assays, we validated that miR-19a-3p fostered the progression of BLCA cells, which is congruous with earlier studies.

By bioinformatics analysis, THBS1 was a possible downstream target of miR-19a-3p, and their binding relationship was verified via dual-luciferase assay. THBS1, a member of the platelet thrombin protein family, has heterogeneity in carrying cancers, which serves not only as an oncogene [24] but also as a tumor suppressor [25]. We disclosed it as a tumor repressor and less expression in BLCA tissues and cells. Yin et al. [25] displayed the repressive role of miR-19a on the THBS1 level, thereby modulating behaviors of colorectal cancer. Italiano et al. [26] indicated that miR-17-92 promotes the formation of angiosarcoma via modulating the THBS1 level. BZRAP1-AS1 hinders the THBS1 level to accelerate liver cancer cell proliferation and migration [27]. We unveiled that overexpression of THBS1 could rescue the promotion impact of miR-19a-3p on malignant behaviors of BLCA cells, consistent with previous research. The above studies suggested that miR-19a-3p could accelerate BLCA cell progression through targeting THBS1.

In conclusion, the forced miR-19a-3p level in BLCA cells could promote the progression of BLCA cells. Meanwhile, miR-19a-3p could inhibit the THBS1 level in BLCA. Moreover, miR-19a-3p exacerbated the malignant progression of BLCA via inhibiting THBS1. We lay the groundwork for miR-19a-3p as a possible target for patients with BLCA. But the study is limited by only one cell line for assays and lacks verification by animal and clinical studies.

## Figures and Tables

**Figure 1:** miR-19a-3p is increased in BLCA. (a) Differential miRNAs in TCGA-BLCA dataset were depicted in a volcano plot (Q1: downregulated miRNAs; Q2: uprequlated miRNAs). (b) miR-19a-3p level in normal tissue and BLCA tissue (blue represents normal tissue, and red represents BLCA tissue). (c) miR-19a-3p level in SV-Huc-1, T24, 5637, and RT4 cell lines detected by qRT-PCR. ^∗^*p* < 0.05.

RETRACTED

**Figure 2:** miR-19a-3p facilitates the malignant progression of BLCA cells. (a) miR-19a-3p level in T24 cells with miR-19a-3p-mimic assayed via qRT-PCR. (b) CCK-8 detected the impact of the forced miR-19a-3p level on proliferation of T24 cells. (c) Impact of the forced miR-19a-3p level on colony formation of T24 cells was detected through colony formation assay. (d) Impact of the forced miR-19a-3p level on migration of T24 cells was assessed via wound healing assay. (e) Transwell invasion assay was used to assess the impact of the forced miR-19a-3p level on T24 cell invasive ability. ^∗^*p* < 0.05.

**Figure 3:** THBS1 is a target of miR-19a-3p. (a) Differential mRNAs in TCGABLCA dataset were depicted in a volcano plot (Q1: downregulated mRNAs; Q2: uprequlated mRNAs). (b) Venn diagram for discovering the target mRNAs of miR-19a-3p. (c) THBS1 level shown in normal tissue and BLCA tissue with blue denoting normal tissue and red denoting BLCA tissue. (d) The expression of THBS1 in SV-Huc-1, T24, 5637, and RT4 cells was assayed through qRT-PCR and Western blot. (e) DLR assay verified the targeted relationship of miR-19a-3p and THBS1. (f) Impact of miR-19a-3p-mimic on the THBS1 level in T24 cells assayed through qRT-PCR and Western blot. ^∗^*p* < 0.05.

**Figure 4:** miR-19a-3p can accelerate malignant behaviors of BLCA cells via binding THBS1. (a) THBS1 level in BLCA cells in three groups was detected through qRT-PCR and Western blot. (b) Proliferation ability of BLCA cells in three groups assayed via CCK-8. (c) Colony formation of BLCA cells in three groups assayed via colony formation assay. (d) Wound healing assay assessed the migratory property of BLCA cells in three groups. (e) Cell invasion assay assessed the invasive property of BLCA cells in three groups. ^∗^*p* < 0.05.

**Table 1:** Primer sequences in qRT-PCR.

Primer	Sequence (5′-3′)
miR-19a-3p	F: CCGTCGGCTTGTTGAGGT
	R: TTCCGTCAGCTCGGAAAGTT
THBS1	F: GCTCCAGTCCTACCAGTGTC
	R: TCAGTCACTTGCGGATGCT
U6	F: AGAGCCTGTGGTGTCCG
	R: CATCTTCAAAGCACTTCCCT
GAPDH	F: CCTGGCCAAGGTCATCCATG
	R: GGAAGGCCATGCCAGTGAGC

## Data Availability

The data that support the findings of this study are available on request from the corresponding author.

## References

[1] Chen W., Zheng R., Baade P. D. (2016). Cancer statistics in China, 2015. *CA: a Cancer Journal for Clinicians*.

[2] Yousef P. G., Gabril M. Y. (2018). An update on the molecular pathology of urinary bladder tumors. *Pathology, Research and Practice*.

RETRACTED

[3] Alfred Witjes J., Lebret T., Compérat E. M. (2017). Updated 2016 EAU guidelines on muscle-invasive and metastatic bladder cancer. *European Urology*.

[4] Siegel R. L., Miller K. D., Jemal A. (2016). Cancer statistics, 2016. *CA: a Cancer Journal for Clinicians*.

[5] Hicks A. M., Chou J., Capanu M., Lowery M. A., Yu K. H., O'Reilly E. M. (2016). Pancreas adenocarcinoma: ascites, clinical manifestations, and management implications. *Clinical Colorectal Cancer*.

[6] Stein J. P., Lieskovsky G., Cote R. (2001). Radical cystectomy in the treatment of invasive bladder cancer: long-term results in 1,054 patients. *Journal of Clinical Oncology*.

[7] Bai R., Cui Z., Ma Y. (2019). The NF-*κ*B-modulated miR-19a-3p enhances malignancy of human ovarian cancer cells through inhibition of IGFBP-3 expression. *Molecular Carcinogenesis*.

[8] Li X., Yan X., Wang F. (2019). Down-regulated lncRNA SLC25A5-AS1 facilitates cell growth and inhibits apoptosis via miR-19a-3p/PTEN/PI3K/AKT signalling pathway in gastric cancer. *Journal of Cellular and Molecular Medicine*.

[9] Zhang B., Liu Y., Zhang J. (2019). Silencing of miR-19a-3p enhances osteosarcoma cells chemosensitivity by elevating the expression of tumor suppressor PTEN. *Oncology Letters*.

[10] Li B., Xie D., Zhang H. (2019). MicroRNA-101-3p advances cisplatin sensitivity in bladder urothelial carcinoma through targeted silencing EZH2. *Journal of Cancer*.

[11] Tsai T. F., Lin J. F., Chou K. Y., Lin Y. C., Chen H. E., Hwang T. I. S. (2018). miR-99a-5p acts as tumor suppressor via targeting to mTOR and enhances RAD001-induced apoptosis in human urinary bladder urothelial carcinoma cells. *OncoTargets and Therapy*.

[12] Song T., Zhang X., Yang G., Song Y., Cai W. (2015). Decrement of miR-199a-5p contributes to the tumorigenesis of bladder urothelial carcinoma by regulating MLK3/NF-*κ*B pathway. *American Journal of Translational Research*.

[13] Zhang C., Ma X., du J. (2016). MicroRNA-30a as a prognostic factor in urothelial carcinoma of bladder inhibits cellular malignancy by antagonising Notch1. *BJU International*.

[14] Chen X., Wu B., Xu Z. (2016). Downregulation of miR-133b predict progression and poor prognosis in patients with urothelial carcinoma of bladder. *Cancer Medicine*.

[15] Wu C. L., Ho J. Y., Hung S. H., Yu D. S. (2018). miR-429 expression in bladder cancer and its correlation with tumor behavior and clinical outcome. *The Kaohsiung Journal of Medical Sciences*.

[16] Morita K., Fujii T., Itami H. (2018). NACC1, as a target of microRNA-331-3p, regulates cell proliferation in urothelial carcinoma cells. *Cancers (Basel)*.

RETRACTED

[17] Chen W., Zhai L., Liu H. (2021). Downregulation of lncRNA ZFAS1 inhibits the hallmarks of thyroid carcinoma via the regulation of miR‑302‑3p on cyclin D1. *Molecular Medicine Reports*.

[18] Sun H. X., Yang Z. F., Tang W. G. (2020). MicroRNA-19a-3p regulates cell growth through modulation of the PIK3IP1-AKT pathway in hepatocellular carcinoma. *Journal of Cancer*.

[19] Fuziwara C. S., Kimura E. T. (2015). Insights into regulation of the miR-17-92 cluster of miRNAs in cancer. *Frontiers in Medicine*.

[20] Lee S., Lee H., Bae H., Choi E. H., Kim S. J. (2016). Epigenetic silencing of miR-19a-3p by cold atmospheric plasma contributes to proliferation inhibition of the MCF-7 breast cancer cell. *Scientific Reports*.

[21] Wa Q., Li L., Lin H. (2018). Downregulation of miR‑19a‑3p promotes invasion, migration and bone metastasis via activating TGF‑*β* signaling in prostate cancer. *Oncology Reports*.

[22] Poli G., Egidi M. G., Cochetti G., Brancorsini S., Mearini E. (2020). Relationship between cellular and exosomal miRNAs targeting NOD-like receptors in bladder cancer: preliminary results. *Minerva Urologica e Nefrologica*.

[23] Yu F. B., Sheng J., Yu J. M., Liu J. H., Qin X. X., Mou B. (2020). MiR-19a-3p regulates the Forkhead box F2-mediated Wnt/*β*-catenin signaling pathway and affects the biological functions of colorectal cancer cells. *World Journal of Gastroenterology*.

[24] Daubon T., Léon C., Clarke K. (2019). Deciphering the complex role of thrombospondin-1 in glioblastoma development. *Nature Communications*.

[25] Yin Q., Wang P. P., Peng R., Zhou H. (2019). MiR-19a enhances cell proliferation, migration, and invasiveness through enhancing lymphangiogenesis by targeting thrombospondin-1 in colorectal cancer. *Biochemistry and Cell Biology*.

[26] Italiano A., Thomas R., Breen M. (2012). The miR-17-92 cluster and its target THBS1 are differentially expressed in angiosarcomas dependent on MYC amplification. *Genes, Chromosomes & Cancer*.

[27] Wang W., Chen G., Wang B. (2019). Long non-coding RNA BZRAP1-AS1 silencing suppresses tumor angiogenesis in hepatocellular carcinoma by mediating THBS1 methylation. *Journal of Translational Medicine*.

